The article "Mechanisms of T-Cell Immunosuppression by Mesenchymal Stromal Cells: What Do We Know So Far?" was published in 2014. Journal: Biomed Res Int.

# Mechanisms of T-Cell Immunosuppression by Mesenchymal Stromal Cells: What Do We Know So Far?

**DOI:** 10.1155/2014/216806

**Published:** 2014-06-16

**Authors:** Rodrigo Haddad, Felipe Saldanha-Araujo

**Affiliations:** ^1^Faculty of Ceilandia, University of Brasilia, 72220-900 Brasilia, DF, Brazil; ^2^Faculty of Health Sciences, University of Brasilia, 70910-900 Brasilia, DF, Brazil

## Abstract

Mesenchymal stromal cells (MSCs) are multipotent cells, which can give rise to several cell types including osteoblasts, adipocytes, and chondroblasts. These cells can be found in a variety of adult and fetal tissues, such as bone marrow, adipose tissue, cord blood, and placenta. In recent years, the biological properties of MSCs have attracted the attention of researchers worldwide due to their potential application for treating a series of clinical situations. Among these properties, special attention should be given to the immunoregulatory potential of those cells. MSCs are able to act on all cells of the immune system, which includes the capacity to inhibit the proliferation and function of T-cells. This feature renders them natural candidates to treat several diseases in which cellular immune response is exacerbated. In this review, we outline the main mechanisms by which MSCs immunosuppress T-cell response, focusing on cell-cell contact, secretion of soluble factors, and regulatory T-cell generation. The influence of surface markers in the immunosuppression process and features of MSCs isolated from different sources are also discussed. Finally, the influences of toll-like receptors and cytokines on the inflammatory microenvironment are highlighted regarding the activation of MSCs to exert their immunoregulatory function.

## 1. Introduction

Bone marrow stromal cells were first described by Friedenstein and coworkers, after the identification of a nonphagocytic cell population with fibroblast-like appearance, able to originate discrete fibroblastic colonies* in vitro* [1, 2]. In 1991, these cells were defined as mesenchymal stem cells (MSCs) by Caplan and regarded as new therapeutic tools for tissue repair, due to their capacity of differentiation and commitment to unique tissue types (e.g., cartilage and bone) [3]. The potential use of MSCs in regenerative medicine approaches to treat diverse diseases has led to a rapid increase in the number of research groups working with those cells. Nevertheless, it also generated several ambiguities and inconsistences in the field, since different terminologies, methods of isolation, expansion, and characterization were reported [4].

In order to solve the discussion concerning the correct nomenclature for these cells [5] and to better describe and define the direction of MSCs research, the Mesenchymal and Tissue Stem Cell Committee of the International Society for Cellular Therapy (ISCT) determined that multipotent mesenchymal stromal cells (with the acronym MSCs) was the more appropriate term to be used. In addition, this committee proposes that these cells must be defined by three minimal criteria. First, these cells must be plastic-adherent when maintained under standard culture conditions. Second, they must present CD105, CD73, and CD90 expression (≥95%) and lack expression of CD45, CD34, CD14, or CD11b, CD79alpha or CD19 and HLA-DR (≤2% positive). Third, they must be able to differentiate into osteoblasts, adipocytes, and chondroblasts when cultured under standard* in vitro* differentiating conditions [4].

The article "Mechanisms of T-Cell Immunosuppression by Mesenchymal Stromal Cells: What Do We Know So Far?" was published in 2014. Journal: Biomed Res Int.

After the identification in a very low percentage in bone marrow (approximately 0.01–0.001% of total mononuclear cells) [3, 6], it was demonstrated that MSCs can be obtained from virtually all adult and fetal human tissues [7]. Furthermore, based on immunophenotypic profile, morphological features, differentiation potential, and gene expression, MSCs are associated with diverse known cell types, very similar to hepatic stellate cells and pericytes and, to a lesser extent, their differentiated “more-restricted” counterparts, as well as fibroblasts. Moreover, MSCs are located in the wall of the vasculature, which could explain the broad distribution throughout the body [7]. Thereby, it is possible to understand the physiologic role of these cells based on the perivascular localization of MSCs. It is believed that they function as a cell repository for tissue repair and could potentially contribute to tissue and immune system homeostasis [7, 8]. In this sense, MSCs possess biological properties extremely attractive to the field of regenerative medicine, such as the ability of MSCs to differentiate into other cell types [9]. In addition, these cells can migrate to damaged or inflamed sites and secrete a variety of bioactive molecules such as cytokines and growth factors. Thereby, by paracrine effects, MSCs display angiogenic, antiscarring, chemoattractant, and immunomodulatory properties [10, 11].

In recent years, the immunosuppressive potential of MSCs has been extensively investigated. This property of MSCs has riveted scientific community attention, especially due to the potential of these cells to treat diseases in which the immune response is exacerbated, such as diabetes and graft-versus-host-disease [12]. Considering the significant advances reported in the field, this review discusses the biology of MSCs, the mechanisms used by these cells to suppress T-cell-mediated immune response, and the recent findings in MSCs activation/licensing.

The article "Mechanisms of T-Cell Immunosuppression by Mesenchymal Stromal Cells: What Do We Know So Far?" was published in 2014. Journal: Biomed Res Int.

## 2. Mechanisms of Immunosuppression

One of the most interesting characteristics of MSCs is the fact that they are hypoimmunogenic. In humans, these cells express low surface levels of major histocompatibility complex (MHC) class I molecules and express neither MHC class II molecules nor costimulatory molecules, such as CD40, CD40L, CD80, and CD86. The expression of MHC class I, although weak, protects MSCs from natural killer (NK) cell-mediated killing; also, the lack of MHC class II expression confers to these cells the ability to escape immune recognition by CD4 cells. Interestingly, both MHC classes I and II molecules can be upregulated by the presence of Interferon *γ* (INF-*γ*), but even in these conditions MSCs do not stimulate immunological response [13–15]. Also, the costimulatory molecule CD40 is upregulated on MSCs under inflammatory conditions [16]. Despite this augment of CD40 expression, T-cells are not full activated because other molecules are required for this activation and the costimulatory system is tightly regulated by inhibitory molecules [17]. For instance, under inflammatory conditions, the inhibitory molecule CD274 (also known by PD-L1) is also upregulated and its expression may be a mechanism used by MSCs to counterbalance the expression of CD40 [16].

In a seminal study, Nicola and coworkers showed that MSCs are able to inhibit T-lymphocyte proliferation in both mixed lymphocyte culture and in the presence of polyclonal activators (interleukin (IL)-2 or Phytohemagglutinin (PHA)). In addition, they demonstrated that both CD4 and CD8 T-cells are equally inhibited by MSCs and that this effect is dose-dependent [18]. These observations lead to a scientific mobilization in order to unravel the mechanisms by which MSCs suppressed T-lymphocyte proliferation. Initially, it was demonstrated that MSCs inhibit proliferation of T-cells proliferation through a MHC-independent mechanism [19]. In addition, MSCs do not induce T-cell apoptosis [20, 21] and the contact T-cells-MSCs leads to T-cell arrest in the G0 phase of cell cycle [22].

Interestingly, some studies suggested that the induction of T-cell suppression by MSCs is dependent, at least in part, on the cross talk between the two cell populations [23]. In addition, the antiproliferative effect of MSCs on the lymphocytes only occurs when these cells are activated, since in a quiescent condition, MSCs support T-cell survival [24, 25]. In fact, it is well known that MSCs do not stimulate T-cell activation. Some studies have shown that MSCs cause a reduction in the expression of activation markers [26, 27], while others found no change in expression of these markers [22, 28].

The article "Mechanisms of T-Cell Immunosuppression by Mesenchymal Stromal Cells: What Do We Know So Far?" was published in 2014. Journal: Biomed Res Int.

Taken together, the ability of MSCs to escape from immune response and to modulate T-cell proliferation renders them attractive candidates for use in cell therapy. The main mechanisms involved in T-cell suppression by MSCs include cell-cell contact, release of soluble factors, and generation of regulatory lymphocytes, which will be discussed more thoroughly below.

### 2.1. Cell-Cell Contact

The first evidence showing that cell-cell contact is necessary for a stronger suppressive effect of MSCs on T-cells was given by Nicola and coworkers [18]. Using a transwell experiment, in which cell-cell contact between MSCs and T-cells was not permitted, the authors showed that even though suppression occurred in such condition, it was much stronger when cells were allowed to have contact. In fact, it was demonstrated that MSCs express integrins (alpha1, alpha2, alpha3, alpha5, alpha6, alphav, beta1, beta3, and beta4), intercellular adhesion molecules (ICAM-1, ICAM-2), vascular cell adhesion protein (VCAM)-1, CD72, and CD58 (LFA-3), among other adhesion molecules on their surface, being able to bind to T lymphocytes with high affinity [29].

Studies exploring the dynamics of contact between MSCs and T-cells are important to understand the behavior of these cells in the inflammatory environment. It seems that, in the first four hours of culture, activated T lymphocytes bind to MSCs and remain trapped for up to 60 h [30]. Interestingly, a study that cultivated adipose-derived MSCs and activated peripheral blood mononuclear cells (PBMC) revealed that this interaction is a specific process, provided that the subset of lymphocytes which interacts with the MSCs is different from the cells that remain in suspension. Moreover, the cellular fraction of T-cells that adhered to MSCs was shown to have an immunosuppressive phenotype [31].

The T-cell attraction process by MSC can be explained by the expression of high levels of several leukocyte chemokines such as chemokine (C-X-C motif) ligand 9 (CXCL9), CXCL10, and CXCL11. The neutralization of CXCR3, a receptor for the T-cell chemokines CXCL9, -10, and -11, reverted immunosuppression by MSCs, revealing the importance of cell adherence in the immune context [32]. In addition to CXCR3, other molecules such as VCAM-1, ICAM-1, and programmed cell death protein 1 (PD-1) have been described to participate in the T-cell suppression by MSCs. In this sense, Ren and coworkers [33] showed that MSCs from mice express high levels of ICAM-1 and VCAM-1 in an inflammatory environment, mediating a close interaction with T-cells. Also,* in vitro* and* in vivo* experiments showed that deletion or blockade of these adhesion molecules lead to a significant reduction in the MSCs-mediated immunosuppression. However, in human MSCs these adhesion molecules did not appear to be crucial for promoting inhibition of T-cell proliferation [34]. In human MSCs, an important mechanism of T-cell suppression involving the cell-cell contact occurs through PD-1 inhibitory molecule and its ligands [35, 36].

The article "Mechanisms of T-Cell Immunosuppression by Mesenchymal Stromal Cells: What Do We Know So Far?" was published in 2014. Journal: Biomed Res Int.

### 2.2. Soluble Factors

Experiments performed with transwell membrane showed efficient suppressive effect against T-cell proliferation, demonstrating that MSCs also exert their immunomodulation by releasing soluble factors [13, 18]. However, the production of suppressive soluble factors is dependent on a cross talk between MSCs and activated T-cells, since the use of supernatants from MSCs culture is not enough for T-cell suppression [27, 36]. On the other hand, supernatants from coculture MSCs-activated T-cell alone can suppress T-cell proliferation [37].

More than thirty soluble factors have been associated with the immunomodulation capacity on T-lymphocyte activation and proliferation by MSCs [38], such as hepatic growth factor (HGF), transforming growth factor-*β* (TGF-*β*) [18], indoleamine 2,3-dioxygenase (IDO) [39], prostaglandin E2 (PGE_2_) [40], nitric oxide (NO) [41], IL-6 [42], IL-10 [43], semaphorin-3A, galectin (Gal)-1 [44, 45], and Gal-9 [46]. Interestingly, some differences are well acknowledged between species. Human MSCs produce IDO to suppress T-cell proliferation, while MSCs from mice exert this function by inducible nitric oxide synthase (iNOS) [47–49]. These functional differences are extremely relevant and should be considered for the interpretation of results obtained by the use of MSCs from mice.

Recently, we have demonstrated an additional mechanism by which MSCs suppress T-cell proliferation [50]. During the cross talk between MSCs and T-cells, there is a production of adenosine by MSCs, which reduce the proliferation of T-cells by signaling adenosine A_2A_ receptor (ADORA2A) on the surface of these cells. Furthermore, a corroborating study showed that MSCs obtained from mice also produce adenosine to suppress T-cell proliferation [51].

Given the complexity of immune system, the combination of synergism and antagonism among these soluble factors released by MSCs should be considered for understanding the immunosuppressive process as a whole [52]. Moreover, there are conflicting results for some mechanisms, but generally these discrepancies can be explained by differences in each study, such as specific features of species, source/tissue of origin, cell isolation method, culture conditions, T-cells : MSCs ratio, and time for data analysis. For instance, Rasmusson and coworkers demonstrated that MSCs-mediated suppression is dependent on the method used to stimulate lymphocytes [53].

The article "Mechanisms of T-Cell Immunosuppression by Mesenchymal Stromal Cells: What Do We Know So Far?" was published in 2014. Journal: Biomed Res Int.

### 2.3. Regulatory T-Cell Generation

Regulatory T-cells (Tregs) are a class of lymphocytes characterized by surface expression of the IL-2 receptor (CD25) and, more specifically, by the presence of high levels of the transcription factor forkhead box P3 (Foxp3). These cells possess the capacity to suppress other immune cells (including T-cells) and can be produced both in the thymus, as a functionally mature subpopulation of T-cells, or induced from naive T-cells in the periphery [54, 55].

When exerting their suppressive effects, MSCs are able to promote the generation of classic CD4^+^CD25^+^Foxp3 Tregs [56, 57]. According to di Ianni and coworkers, MSCs can act as a potential “homeostatic niche” for Tregs, since they recruit, regulate, and maintain T-regulatory phenotype and function over time [57]. Moreover, MSCs possess ability to expand Tregs through a mechanism dependent on human leukocyte antigen G (HLA-G) 5, a nonclassic HLA-G [58]. Given the possibility of using these cells for cell therapy, the* in vitro* production of Tregs became of great relevance [59, 60]. Although Tregs therapy holds great promise, there is a major point to be considered: the stabilization of Foxp3 expression, since a fraction of expanded Tregs loose Foxp3 expression and consequently their suppressive potential. Furthermore, some of the T-cells convert back into effector cells and could exert pathogenic functions [61, 62].

Several studies have been conducted in order to describe the mechanisms by which MSCs generate Tregs. In part, this process occurs initially by a nonredundant contribution that involves MSC-derived PGE_2_, TGF-*β*1, and cell-cell contact [63]. Furthermore, it has been demonstrated that, during the coculture with T-cells, MSCs secrete leukemia inhibitory factor (LIF) and antibody blockage of this protein leads to decreased Foxp3 positive regulatory T-cells [64, 65]. A recent study showed that the activation of Notch-1 pathway in CD4^+^ T-cells induces Treg differentiation, since MSCs express the Notch 1 ligands Jagged1, Jagged2, and Delta-Like (DLL) 1, 3, and 4 [66]. Another study showed that MSCs produce heme oxygenase-1 (HO-1), which is important to IL-10-producing Treg (Tr1) generation by a mechanism that remains elusive [67, 68]. In this sense, it is important to note that IL-10 secretion by Tr1 may be crucial to HLA-G5 production by MSCs, and consequently to Treg expansion [58]. Recently, a coculture MSCs-PBMC study showed that monocytes are essential for Tregs induction by MSCs. In the same study, it was demonstrated that MSCs sustained the differentiation of monocytes into macrophage type 2 cells, which secrete CCL 18 and IL-10. This process contributes indirectly to Treg generation [69]. Interestingly, MSCs are also capable of inducing the generation of different lymphocyte subtypes with regulatory phenotypes [70]. In this sense, our group demonstrated that, in coculture conditions, MSCs induce a shift from canonical to noncanonical NF-*κ*B signaling in T-lymphocytes, leading these cells to sustain the expression of CD69 [71] as an immune suppressive marker [72, 73].

The article "Mechanisms of T-Cell Immunosuppression by Mesenchymal Stromal Cells: What Do We Know So Far?" was published in 2014. Journal: Biomed Res Int.

Recently, an important finding was reported by Yan and colleagues [74]. Using a coculture system, they showed that MSCs are able to enhance the suppressive potential of Tregs by promoting an upregulation of PD-1 on these cells. Besides promoting the generation of Tregs with high suppressive potential, MSCs possess ability to expand Tregs. As commented above, this process is, in part, dependent on human leukocyte antigen G (HLA-G) 5, a nonclassic HLA-G [58]. When at low concentrations, by a mechanism apparently dependent on IL-6, MSCs are able to support T-cell proliferation. Among these cells in expansion, Tregs are found [42].

Although MSC-derived PGE_2_ plays a role in the Tregs proliferation as cited above [63, 75], this molecule also prevents the differentiation of naive T-cells into proinflammatory Th17 cells. Also, MSCs act directly on Th17 cells promoting the differentiation of these cells into Tregs. Under inflammatory conditions, MSCs are able to mediate the adhesion of proinflammatory Th17 cells via chemokine receptor 6 (CCR6) and induce the conversion of these cells into functional Treg cells Foxp3^+^ [76]. Interestingly, Lee and colleagues [77] recently reported that MSCs promote an upregulation of CD39 on Th-17 cells inhibiting the function of these cells by adenosine production. Although these cells have not been functionally tested, the fact that CD39 is a marker of Tregs [78, 79] suggests that, like CCR6, adenosine could promote a shift from Th-17 cells into Tregs.

Finally, although several evidences have demonstrated that MSCs generate Tregs to modulate T-cell proliferation* in vitro*,* in vivo* studies showed that the contribution of this mechanism for the suppressive effect of MSCs is controversial [80, 81]. It would be important to conduct studies with isolated Tregs generated by MSCs in order to better understand the contribution of each cell type to the suppression of T-cell proliferation.

## 3. MSCs from Different Sources: Do They Share the Same Features?

As mentioned above, MSCs can be isolated from a variety of adult and fetal tissues, including dental pulp [82], adipose tissue [83], skin [84], cord blood [85], liver [86], synovium [87], pancreas [88], lung [89], placenta [90], amniotic fluid [91], and peripheral blood [92].The use of different sources of MSCs was motivated by several reasons: first, the use of ethically approved sources which otherwise would be discarded in hospitals (e.g., placenta and lipoaspirate) and, second, the scientific advance regarding the characterization of MSCs from other tissues than bone marrow, assessing whether the immunosuppressive property is also a feature of these MSCs. Third, the use MSCs obtained from bone marrow exposes the donor to a painful and invasive procedure, leading to the use of noninvasive and ethically nonproblematic sources.

The article "Mechanisms of T-Cell Immunosuppression by Mesenchymal Stromal Cells: What Do We Know So Far?" was published in 2014. Journal: Biomed Res Int.

Commonly designed as a gold standard, bone marrow derived MSCs (BM-MSCs) are the most investigated cell type [93]. Instead, MSCs from placenta (Pl-MSCs), umbilical cord (UC-MSCs), Wharton's jelly (WJ-MSCs), and adipose tissue (AT-MSCs) are also used in studies, considering their known immunosuppressive potential [94–102]. In addition, several works showed that MSCs obtained from other tissues, including lung, spleen, thymus, and others, also possess capacity to suppress T-cell proliferation [31, 97, 102–107]. Although sharing basic biological properties, MSCs may present specific favorable features depending on the source from which they were obtained, such as expansion potential and frequency. For instance, AT-MSCs and Pl-MSCs allow obtaining a large number of cells with high expansion potential; the umbilical cord is also an excellent tissue for MSCs isolation; in contrast, the easy and risk-free availability of umbilical cord blood as a tissue for MSCs isolation is negatively counterbalanced by the lower yields of MSCs from this source [90, 108, 109]. Regarding the biological features, MSCs from different tissues may differ even when isolated from the same donor. Recently, it was demonstrated that MSCs from dental pulp and periodontal ligament of the same donor have distinct mesenchymal properties, including differences on multipotentiality, immune parameters, and response to proinflammatory cytokines [110].

Considering the immunosuppressive potential of MSCs, some studies investigated the differences between BM-MSCs and MSCs isolated from other tissues. In this sense, a study with MSCs isolated and expanded from adult human tissues, including AT-MSCs, UC-MSCs, and WJ-MSCs, showed that these cells presented a pattern of surface markers expression typical of BM-MSCs. In addition, all non-bone marrow populations suppressed mitogen-induced T-cell proliferation at levels comparable with BM-MSCs, and, at least in part, by similar mechanisms [99]. In another report, WJ-MSCs and AT-MSCs presented a higher suppressive capacity compared to BM-MSCs, regardless of the stimuli used to activate T-cells (cellular or mitogenic stimuli). Furthermore, WJ-MSCs and AT-MSCs showed faster proliferation and greater expansion capabilities compared to BM-MSCs [96]. An interesting fact is that, if this proliferative advantage also occurs in inflammatory environments, this biological behavior could partially explain the greater suppressive potential of these cells by a numeric condition.

The article "Mechanisms of T-Cell Immunosuppression by Mesenchymal Stromal Cells: What Do We Know So Far?" was published in 2014. Journal: Biomed Res Int.

Another comparative study showed that Pl-MSCs are immunophenotypically similar to BM-MSCs but exhibit a stronger suppressive potential against either mitogen or alloantigen stimulated T-cells. This finding might be explained by the source of cells, since the placenta is an immunologically privileged site that supports the maternal-fetal tolerance [101]. In contrast, another study showed that BM-MSCs and umbilical cord blood-derived MSCs (UCB-MSCs), but not Pl-MSCs, significantly inhibited the proliferation of both CD4^+^ and CD8^+^ activated T-cells by cell-cell contact, favoring the generation of regulatory T-cells subsets, and producing the increase of IFN-*γ*, IL-10, and PGE_2_ [111]. It is important to note that placenta is an organ that possesses different regions, such as amniotic epithelial, amniotic mesenchymal, chorionic mesenchymal, and chorionic trophoblastic. Therefore, several cell types can be obtained depending on the chosen region. This complexity becomes important to the standardization of cell isolation methods from this tissue. Depending on the isolated cell type, the interpretation of comparative studies may be misleading [112]. Recently, an important finding was shown by di Trapani and colleagues. Analyzing the suppressive potential of stem cells from different tissues—BM-MSCs, olfactory ecto-MSCs, non-MSCs leptomeningeal stem cells, and human c-Kit-positive stem cells isolated from the amniotic fluid, adult heart, and adult lung, they demonstrated that the capacity to modulate the immune response is not an exclusive property of MSCs, but a common feature of all stem cells evaluated [113].

Certainly, there is considerable truth in the studies of MSCs immunosuppression. Nevertheless, there are some conflicting data, even though the population diversity of the primary cultures as well as the tissue- and species-origin of the MSCs can justify the inconsistencies presented by some studies [109]. Despite such discrepancies, the knowledge that the suppressive potential of BM-MSCs is a property shared by MSCs from other tissues and by other stem cells is of importance for the establishment of new alternatives for the clinical use.

The article "Mechanisms of T-Cell Immunosuppression by Mesenchymal Stromal Cells: What Do We Know So Far?" was published in 2014. Journal: Biomed Res Int.

## 4. MSCs Surface Markers and Their Influence on Immunosuppression

Despite the standardization of requirements according to Mesenchymal and Tissue Stem Cell Committee of the ISCT to define MSCs, data from many studies remain heterogeneous. In part, this heterogeneity occurs because there is no consensus on a specific surface marker for these cells, which would allow obtaining a pure and homogeneous cell population. As cited previously, MSCs from different sources may present distinct features, which also include the expression of certain surface markers according to the tissue from which they were obtained. These differences render establishing a definitive marker for MSCs very difficult. For instance, the expression of CD271 is present on BM-MSCs and on MSCs from synovium, but not on Pl-MSCs [114–116]. The expression of CD34, a typical marker of hematopoietic stem/progenitor cells, is present on AT-MSCs [117–119] and in a fraction of BM-MSCs [120, 121].

The expression of surface markers on MSCs is also influenced by cultivation time. The expression of CD34 on AT-MSCs disappears when these cells are propagated in culture [122]. Likewise, the number of STRO-1-positive BM-MSCs progressively declines during prolonged culture [123]. On the other hand, the expression of other markers on AT-MSCs, such as CD73, CD90, and CD166, increases during progressive stages of passage [122].

Interestingly, some surface markers have been associated with immunosuppressive capacity of MSCs. Stro-1 positive BM-MSCs inhibited PBMCs proliferation more efficiently than heterogeneous BM-MSCs [124]. However, it is important to note that the initial percentage of STRO-1 positive cells in the MSCs population was only 6%. This low yield can be a limiting factor for the clinical use of these STRO-1 enriched cells. Similarly, the absence of CD90 molecules may be related to loss of MSCs immunosuppressive potential. This surface marker appears to be involved in the control of soluble HLA-G and IL-10 production, both involved in immunosuppression process [125]. The CD271 positive BM-MSCs also possess a privileged immunosuppressive capacity. These cells induce an expansion of naïve Tregs, which in part, can be responsible for the potent suppressive effect [126]. In this line, VCAM-1-enriched MSCs possess high immunomodulation activity [127]. This is not surprising, since there is a high expression of this marker on the surface of MSCs and the suppressive role of VCAM-1 on MSCs is well defined, as discussed above. Likewise, CD39 and CD73 double positive MSCs also appear to have a potent suppressive potential. As demonstrated by our group, these surface markers are upregulated in inflammatory environments and induce adenosine production, which in turn, contributes to T-cell immunosuppression [50].

The article "Mechanisms of T-Cell Immunosuppression by Mesenchymal Stromal Cells: What Do We Know So Far?" was published in 2014. Journal: Biomed Res Int.

Taken together, these studies show that surface markers effectively participate in immunosuppression mechanism exerted by MSCs. The obtention of cell populations with higher expression of these molecules could be an alternative to improve the efficiency of MSC-mediated inhibition of T-cell proliferation.

## 5. Mesenchymal Stromal Cells “Activation”

Several studies have shown that MSCs not only possess immune-modulatory capacity, but also antiapoptotic properties and supporting activity toward different cell types [128] under resting conditions. MSCs are able to regulate the survival, self-renewal, migration, and differentiation of hematopoietic stem cells (HSC) through several mechanisms including cell-cell contact and soluble factors [129]. Also, MSCs support the development of B cells from HSCs [130]. Moreover, the proliferation and differentiation into immunoglobulin-secreting cells of all peripheral B-cell subsets are influenced by MSCs [131]. On the other hand, other studies showed that MSCs block the proliferation and differentiation of B cells, but they also increase B-cell viability [132]. MSCs also influence T-cell behavior, supporting T-cell survival in a quiescent state, when they are subjected to stress conditions, which could lead to apoptosis [25]. In addition, antigen-presenting cell (APC) property and proinflammatory activity are also shared by MSCs [133, 134]. Furthermore, there are evidences that MSCs support tumoral progression through mechanisms that include signaling networks with other cells of tumor microenvironment [135, 136], tumoral angiogenesis [137–139], cellular alteration by hybrid/chimeric cell generation [140, 141], cancer growth by promoting the proliferation and migration of MSCs themselves [142], and metastasis induction [143–145]. Unlike this protumorigenic activity, there are also growing evidences showing that human MSCs exert antitumorigenic responses in the tumor sites [146, 147] possibly by the inhibition of the Wnt signaling pathway [148, 149] and inhibition of the Akt signaling pathway [150], both important pathways in the tumor development and progression [151, 152]. Taken together, these findings strongly suggest that the immunomodulatory capacity of MSCs is not constitutive.

In the last few years, it has been proposed that MSCs could be polarized into two homogenously acting phenotypes, classified as MSC1 and MSC2 according to the stimulation of specific toll-like receptors. While MSC1 have proinflammatory and immunocompetent phenotypes, MSC2 possess immunosuppressive properties [153]. Furthermore, other studies have shown that environmental inflammatory cytokines, such as INF-*γ*, tumour necrosis factor (TNF)-*α*, and IL-1 *α*/*β*, are necessary to “license” the MSCs to exert or improve their immunosuppressive actions [154]. In this sense, studies have shown that proinflammatory cytokines promote differential regulation of MSCs immunomodulatory factors, including IDO, PGE_2_, TGF-*β*, TSG-6, and NO [32, 155]. Therefore, MSCs depend on a complex cross talk with several elements to inhibit the effector functions of T lymphocytes.

The article "Mechanisms of T-Cell Immunosuppression by Mesenchymal Stromal Cells: What Do We Know So Far?" was published in 2014. Journal: Biomed Res Int.

### 5.1. Interferon-Gamma (INF-*γ*)

Produced by natural killer (NK) and natural killer T (NKT) cells during innate immune response, INF-*γ* is an important cytokine involved in the regulation of both immune and inflammatory responses. It stimulates the activation and differentiation of several cell types including the generation of T helper (Th)1 from CD4^+^ cells [156]. During the adaptive immune response, both activated CD4^+^ and differentiated Th1 cells produce large amounts of INF-*γ*, providing effective protection against intracellular pathogens [157].

On the other hand, studies have shown that, in the presence of MSCs, INF-*γ* leads to the suppression of T-cell proliferation. This effect is exerted by immunoregulatory machinery of MSCs, since inhibition of INF-*γ* receptor of these cells reverts this effect [20]. In this line, MSCs lacking INF-*γ* receptor do not possess immunosuppressive activity against T-cell proliferation [32]. Corroborating such observation, a strong inhibition of MSCs growth was recently demonstrated following the addition of preactivated lymphocytes, but not after adding resting T-cells. Conversely, the licensing with IFN-*γ* partially protected MSCs from preactivated lymphocytes [158]. The effect of INF-*γ* in MSCs licensing can also be observed* in vivo*. MSCs pretreated with INF-*γ* are able to abrogate graft versus host diseases (GvHD) more efficiently than nontreated MSCs. Furthermore, when administered during bone marrow transplantation, INF-*γ*-treated MSCs prevent mortality from GvHD [159]. Thus, INF-*γ* is an essential factor to licensing (or priming) MSCs to exert their immunoregulatory functions against T, B, and NK cells [128].

Up to now, all signaling pathways involved in the licensing by INF-*γ* are unknown, but there are evidences that the increase of soluble factors and receptors related to immunosuppression mechanisms is involved. Some authors described that INF-*γ* activates the synthesis and transcription of IDO-1 and augments the expression of hepatocyte growth factor (HGF) and TGF-*β* by MSCs [20, 160]. Likewise, human AT-MSCs, which also possess immunoregulatory activity, require the INF-*γ*-mediated IDO-1 to modulate immune responses [161].

The article "Mechanisms of T-Cell Immunosuppression by Mesenchymal Stromal Cells: What Do We Know So Far?" was published in 2014. Journal: Biomed Res Int.

Another molecule related to INF-*γ* signaling is Galectin (Gal)-9, which was shown to be released by MSCs upon stimulation with INF-*γ*. There are evidences that Gal-9 is involved in the immunosuppression activity by a mechanism not elucidated so far, since MSCs with Gal-9 knockdown loose a significant portion of their antiproliferative effects on T-cells [46]. Also, INF-*γ* acts directly on MSCs leading to increased levels of programmed death ligand 1 (PD-L1, also called B7H1) and 2 (PDL-2, also called B7DC) in their surface, inhibiting effector T-cell function through the ligands of PD-1. Furthermore, the increase of these inhibitory molecules on the surface of MSCs supports the importance of cell-cell contact mechanisms in MSC-mediated immunosuppression [35, 162]. Finally, INF-*γ* allows MSCs to survive in the inflammatory environment. This is a result of the resistance acquired by MSCs against activated NK-mediated attack after INF-*γ* stimulation [163]. Despite the fact that the action of INF-*γ* in the licensing of MSCs is well known, the concentration of this inflammatory cytokine appears to be important, since low levels of INF-*γ* stimulate APC function on MSCs and exerts proinflammatory effect [133, 164, 165]. However, the local production of INF-*γ* in the* in vivo* microenvironment cannot be measured [128]. Thus, the INF-*γ* levels used for MSCs licensing should be evaluated carefully for clinical applications.

### 5.2. Other Proinflammatory Cytokines

It has been published that INF-*γ* activates the immunoregulatory functions of MSCs concomitantly with other proinflammatory cytokines, such as TNF-*α*, IL-1*α*, or IL-1*β* [32, 128, 155, 161]. The vast majority of studies showed that, when used as single agents, these cytokines are unable to trigger the inhibition of T-cell proliferation by MSCs. However, the use of INF-*γ* with one of the other cytokines enhances the immunomodulatory effect of MSCs compared to INF-*γ* alone. In this line, the use of antibodies to block all these cytokines (INF-*γ*, TNF-*α*, and IL-1*α*/*β*) abolishes the immunoregulatory function of MSCs against T-cell proliferation in a superior manner compared to the use of anti-INF-*γ* alone. In the same system, the use of antibodies to block single cytokines did not obliterate the inhibition of T-cell proliferation by MSCs [32].

TNF-*α*, a proinflammatory cytokine secreted by T-cells, NK, cells and macrophages, induces the expression of several proteins related to immunoregulation and increases the capacity of migration of MSCs [166–168]. A study recently demonstrated that, before suppressing T-cell proliferation, MSCs increase the early production of IFN-*γ* and IL-2 by CD3/CD28-activated PBMCs. After treatment with TNF-*α* and IFN-*γ*, MSCs were less effective at increasing proinflammatory cytokine production by activated PBMCs and more efficient at inhibiting T-cell proliferation [169]. Studies also showed that use of TNF-*α* associated with INF-*γ* promotes increase of HGF, PGE_2_, and COX-2 levels by MSCs, favoring the inhibition of T-cell proliferation [155]. Furthermore, secretion of superoxide dismutase 3 (SOD3) by human BM-MSCs is regulated synergistically by TNF-*α* and INF-*γ* [170]. In turn, SOD3 appears to be involved in the inhibition of T-cell activation and proliferation [171]. Moreover, treatment of MSCs with TNF-*α* and INF-*γ* changes the microRNA profile, indicating that the participation of these small molecules in the immunosuppressive capacity of MSCs. With this in mind, it was recently demonstrated that microRNA (miR)-155 inhibits the immunosuppressive capacity of MSCs by reducing iNOS expression and thereby NO release [172]. Finally, TNF-*α* and INF-*γ* act concomitantly in the induction of chemokines involved in the chemotaxis and the inhibition of immune effector cell proliferation, such as CCR5, CCR10, CXCL9, CXCL10, and CXCR3 [32, 173].

The article "Mechanisms of T-Cell Immunosuppression by Mesenchymal Stromal Cells: What Do We Know So Far?" was published in 2014. Journal: Biomed Res Int.

In contrast to other studies, very recently it has been shown that TNF-*α* alone is also enough to upregulate the chemokine CXCR4 in human bone marrow-derived MSCs in a time- and dose-dependent manner [174]. Some authors suggest that lower expression of CXCR4 by MSCs lead to the failure of these cells to migrate into inflammation site and consequent loss of immunoregulatory functions [175]. Also, other authors showed that TNF-*α* released by activated T-cells confers immunoregulatory properties upon MSCs by binding to TNF-receptor 1 (TNF-R1) and activating the nuclear factor kappa B (NF-*κ*B) pathway [176, 177], contrasting with other studies, in which INF-*γ* seems to be a required factor. Besides, the presence of APRIL and BAFF—two TNF family proteins—is able to modulate the functionality of MSCs through activation of extracellular signal-regulated kinases 1/2 (ERK1/2) and Akt kinases. They increase the proliferation of MSCs without changing the immunomodulatory properties of these cells [178].

The IL-1 family of cytokines, which includes IL-1*α* and IL-1*β*, exerts a crucial role as mediator of the inflammatory response, playing an important part in the body's natural responses and the development of pathological conditions leading to chronic inflammation [179].* In vitro* studies showed that the full T-cell suppressive ability of MSCs requires the production of IL-1*β* by monocytes. In turn, IL-1*β* enhances the secretion of TGF-*β* by MSCs, which is involved in the inhibition of T-cell proliferation [26]. Other study showed that, in the presence of INF-*γ*, either TNF-*α* or IL-1*α* induces the expression of ICAM-1 and VCAM-1. These adhesion molecules are also essential for MSCs-mediated immunosuppression [33]. In addition, the immunomodulatory capacity of MSCs is activated by concomitant stimulus of INF-*γ* and IL-1*α* or IL-1*β*. These combinations induce the upregulation of nitric oxide synthase (NOS), which catalyzes the production of NO, as well as several leukocyte chemokines that may bring immune cells, including T-cells, into close proximity of MSCs. High levels of NO can suppress T-cell proliferation [32]. More recently, it was observed that both IL-1*α* and IL-1*β* alone induce the expression of Gal-9. The same study also showed that upregulation of Gal-9 was functionally important and contributed to the immunosuppressive effects of MSCs [46].

The article "Mechanisms of T-Cell Immunosuppression by Mesenchymal Stromal Cells: What Do We Know So Far?" was published in 2014. Journal: Biomed Res Int.

### 5.3. Toll-Like Receptors

Toll-like receptors (TLRs) are type I membrane proteins expressed either in the plasma membrane or intracellularly by immune or nonimmune cells. Most mammalian species have 10 to 15 subtypes of TLRs; while humans possess 10 of them, mice possess 12 subtypes. Each TLR recognizes and is activated by a small collection of molecules derived from pathogens. TLRs act mainly to initiate an innate immune response against invading microbes and, through dendritic cells, activate the adaptive immune response to recognize specific pathogens [180]. Interestingly, MSCs also express some TLRs at the protein level, including TLR2, TLR3, TLR4, TLR7, and TLR9. The ligand-mediated triggering of some TLRs may control the proliferation and differentiation of MSCs [181–183].

The implication of TLRs on immunomodulatory activity of MSCs has also been reported [153, 184–186]. The stimulation of TLR2 impairs the capacity of MSCs to inhibit the lymphocyte proliferation and promotes the decreasing of the generation of CD4^+^CD25^+^FOXP3 Tregs. In the same study, TLR4 stimulation had no effect on T-cell proliferation or Tregs generation [187]. The stimulation of TLR3 and TLR4 on MSCs induces the downregulation of Notch ligand Jagged-1 on these cells and the consequent reduction of their suppressive activity on T-cell proliferation [184]. In line, the stimulation of TLR3 and TLR4 in MSCs promotes the inflammatory response against pathogens by increasing the expression of several proinflammatory cytokines, including IL-1, IL-6, IL-8, TNF-related apoptosis inducing ligand (TRAIL), and CCR5, as well as enhancing the activity of iNOS [185]. Moreover, preactivation of MSCs with TLR3 or TLR4 ligands reduced production of HGF and PGE2, decreasing their capacity to inhibit T-cell proliferation [188]. On the other hand, the same author showed that the source of MSCs influences their TLRs profiles as well their functional properties. In this study, triggering TLR3 or TLR4 on MSCs from bone marrow, adipose tissue, and Wharton jelly's did not impair the immunosuppressive capacity of these cells [188]. Furthermore, a study showed that the stimulation of TLR3 and TLR4 before the coculture with T-cells enhances the immunomodulatory capacity of MSCs through the indirect induction of IDO1 [186]. MSCs from dental pulp and dental follicle are also able to inhibit T-cell proliferation* in vitro*, and this effect is potentiated by TLR3 activation. The same study showed that TLR4 activation increased the potential of immunomodulation of dental follicle MSCs, but decreased it in dental pulp MSCs [189]. Finally, the prestimulation of TLR4 or TLR5 did not affect the immunomodulatory activity of UCB-MSCs [190].

The article "Mechanisms of T-Cell Immunosuppression by Mesenchymal Stromal Cells: What Do We Know So Far?" was published in 2014. Journal: Biomed Res Int.

As shown above, conflicting results in the literature have been reported regarding the immunomodulation of TLR-stimulated MSCs. Waterman and collaborators proposed a model that could explain these contradictory results. They hypothesized that, in parallel with macrophage polarization, two different types of MSCs with distinct phenotypes could be generated after TLRs stimulation. TLR4-stimulated MSCs released proinflammatory cytokines, such as IL-6, IL-8, or TGF-*β* (MSC1 phenotype). By contrast, TLR3-primed MSCs produced anti-inflammatory molecules such as IL-4, IDO, or PGE_2_ (MSC2 phenotype). While MSC1 activated T-cells, MSC2 maintained the capacity to inhibit lymphocyte proliferation. These results were obtained in a low level and short-term TLR-priming protocol. Thus, the licensing process of MSCs toward either MSC1 or MSC2 phenotypes depends on the TLR-ligand concentration, timing, and kinetics of activation [153]. Due to the fact that the effects of TLRs ligands on MSCs immunoregulatory functions are still confusing [153, 184, 186, 188], further investigation is required to clarify the role of TLRs in the process of MSCs licensing.

## 6. Concluding Remarks

Despite years of research, culture-expanded MSCs* in vitro* did not become a widely prescribed therapeutic agent for diseases in which cellular immune response is exacerbated. To date, numerous cell based-therapy employing MSCs against autoimmune diseases have been registered at clinicaltrials.gov. Although the infusion of MSCs appears to be safe and well tolerated, there are some conflicting results related to the clinical outcomes. In addition, some studies are not finalized yet. Increasingly substantial progress has been made in our understanding of the interactions between MSCs and immune cells. The meticulous understanding of both the immunoregulatory mechanisms and MSCs licensing by different stimuli is essential; the use of MSCs from suitable sources with appropriated biological features for each specific case could favor the clinical outcome after MSCs-based autoimmune therapy; also,* in vitro* conditioning by cytokine exposure and/or TLRs stimulation prior the use* in vivo* could boost the effectiveness of MSCs. Despite the large amount of data obtained so far, it is still necessary to acquire new knowledge about the complex cross talk between MSCs and the immune system, in order to allow for the wide and effective use of MSCs in clinical settings.
